This article has been retracted.

# IoT-Based Wearable Sensors and Bidirectional LSTM Network for Action Recognition of Aerobics Athletes

**DOI:** 10.1155/2021/9601420

**Published:** 2021-07-26

**Authors:** Jing Ye, Hui Wang, MeiJie Li, Ning Wang

**Affiliations:** ^1^School of Sports Science, Tianjin Normal University, Tianjin 300387, China; ^2^Sports Institute, Henan Agricultural University, Zhengzhou 450002, China; ^3^Faculty of Physical Culture, Gdansk University of Physical Education and Sport, Gdansk 80-336, Poland; ^4^Sports Institute, Korea Gangneung-Wonju National University, Gangneung 25457, Republic of Korea

## Abstract

Aerobics is the fusion of gymnastics, dance, and music; it is a body of a sports project, along with the development of the society. The growing demand for aerobics inevitably increases the demand for aerobics coach and teacher and has opened elective aerobics class which is an effective way of cultivating professional talents relevant to aerobics. Aerobics has extended fixed teaching mode and cannot conform to the development of the times. The motion prediction of aerobics athletes is a new set of teaching aid. In this paper, a motion prediction model of aerobics athletes is built based on the wearable inertial sensor of the Internet of Things and the bidirectional long short term memory (BiLSTM) network. Firstly, a wireless sensor network based on ZigBee was designed and implemented to collect the posture data of aerobics athletes. The inertial sensors were used for data collection and transmission of the data to the cloud platform through Ethernet. Then, the movement of aerobics athletes is recognized and predicted by the BiLSTM network. Based on the BiLSTM network and the attention mechanism, this paper proposes to solve the problem of low classification accuracy caused by the traditional method of directly summing and averaging the updated output vectors corresponding to each moment of the BiLSTM layer. The simulation experiment is also carried out in this paper. The experimental results show that the proposed model can recognize aerobics effectively.

## 1. Introduction

In the current era, aerobics [1, 2] is a popular sport around the world. The special aerobics course aims to train aerobics teachers or professionals with excellent aerobics skills and teaching ability. However, at the moment, most colleges and universities have started special aerobics classes and continue the traditional teaching model. The students are learning calisthenics skill content and its way in a relatively closed category. The traditional calisthenics teaching cannot comply with the demand of the current period of aerobics. So, colleges and universities need to optimize aerobics teaching methods [3–5], innovate teaching mode, and find a new direction for sports teaching ideas. Aerobics combines gymnastics [6–8], dance [9,10], music [11], and other elements, which can cultivate students' artistic aesthetic ability and promote the development of students' physical quality [12]. Aerobics can improve the body's functional level and contribute to the human body's resistance to disease. Long-term aerobics can also yield a better body shape. Calisthenics has a variety of sports, promotes the development of the national fitness movement, and is a relatively considerable degree of popularity of a sport. Aerobics has become a professional course in schools, and more and more students are fond of this sport. Aerobics teaching courses in various colleges and universities are set up as elective, compulsory, and special courses according to the requirements of the new curriculum reform. Aerobics elective courses are mainly aimed at students who are not majoring in physical education.

The main training objectives are to develop physical fitness and cultivate interest. The required course of aerobics is aimed at the students majoring in physical education. Its training goal is to train students to have specific aerobics skills. The students of the aerobics class aim to train the aerobics professional and technical talents. With the development of society and the increasingly fierce social competition, the cultivation of students needs to conform to the changes of the current times and keep pace with the times. Students are required to learn basic calisthenics skills and consider the needs of students' future careers. The current aerobics special courses mostly use the traditional teaching model. With the development of time, students will feel that learning is boring, learning enthusiasm is not high, and the learning efficiency of technical movements is low. With the development of society and new curriculum reform requirements, aerobics' teaching materials and teaching have higher requirements. The teaching content needs to be gradually enriched, and the teaching methods need to keep pace with the times. The current trend of aerobics project development is to absorb excellent teaching methods or apply advanced teaching tools to traditional aerobics professional courses and promote teaching effectiveness.

As a set of new teaching aids, the IoT-enabled wearable inertial sensor [13–15] and the BiLSTM network aerobics action recognition system not only combine the advantages of IoT and inertial sensor but also adds the neural network action recognition [16, 17] module, which is not only in a novel form. An aerobics project can make up for any shortcomings in traditional teaching and enhance students' interest in aerobics and course participation. The research of this system is beneficial to the scientific development of aerobics and other sports in the future.

The main contributions of this paper are as follows:

1. The IoT-based wearable inertial sensor and BiLSTM network aerobics action recognition model enrich the conventional aerobics teaching methods. It makes up for the deficiency of conventional teaching, provides a theoretical basis for the development of innovative aerobics teaching methods, and provides a theoretical basis for optimizing professional aerobics courses.
2. By combining the attention mechanism on the BiLSTM network, we solve the problem that the traditional method directly sums up the updated output vectors corresponding to each moment in the BiLSTM layer. It takes the average value, which leads to low classification accuracy, to improve the robustness of the aerobics action recognition model.

The rest of the paper is organized according to the following pattern. In Section 2, the background study is given. In Section 3, the methodology is discussed. The experiments and results are elaborated in Section 4. Finally, Section 5 concludes the paper.

## 2. Background

### 2.1. Aerobics

Aerobics originated in 1968 from the space agency. In 1969, Jackie Solon defined aerobics as a combination of gymnastics and modern dance. The famous Swedish modern gymnast Meekman defined aerobics as “the rhythmic body movement into the gymnastic movements, which can not only reflect the creativity of movements but also conform to the progress of the times as a new form of gymnastics.” Masako Sato wrote “self-taught calisthenics” and opened the first calisthenics school in Japan in 1980, defining calisthenics as “the application of effective movements from jazz techniques to body movements, using the principles of gymnastics as part of gymnastics.”

### 2.2. The Current Situation of Aerobics Teaching

The popularization of aerobics teaching in various colleges and universities makes more students understand and love the aerobics movement. However, with the progress of the times, there are many problems in aerobics teaching, so each scholar has analyzed the aerobics teaching differently. Fan Yang, a scholar, thoroughly analyzed aerobics' teaching situation in colleges and universities in Beijing from teaching content and teaching methods. The primary deficiencies in aerobics teaching are analyzed: the students' lack of understanding and understanding of aerobics class causes the students to be not optimistic about aerobics learning and makes the teaching quality and efficiency of aerobics' more efficient courses are not high. The calisthenics teaching materials are old and mostly self-compiled. There is no scientific and complete teaching system, making it a stumbling block to the development of calisthenics. Only the reform can comply with the development needs of calisthenics. The teaching content is single and lacks innovation. There is no precise stage, and the teaching knowledge is simple, which cannot meet the current teaching show. At present, many colleges and universities use multimedia equipment or new forms in calisthenics teaching, but they generally use conventional calisthenics teaching.

At present, many scholars have carried out much research on the teaching mode of aerobics, aiming to make up for the shortcomings of the traditional teaching mode [18]. Among them, Fang Ting, a scholar, studied the application of “five-star teaching mode” in aerobics courses through literature and teaching experiment. It is found that the traditional teaching mode of aerobics plays a significant role in exerting the leading role of teachers and systematically carrying out the teaching of technical movements. With the gradual development of aerobics project, the problems in conventional teaching are increasingly prominent: the single teaching method, too much attention to the teaching of technology, and neglect of students' independent learning ability and students' psychological needs, resulting in students' learning enthusiasm is not high. Therefore, to stimulate the degree of participation of students in learning is the main task. Therefore, it is very important to accurately identify and evaluate aerobics movements [19–23] to assist teaching so that students can learn movement routines faster, stimulate their learning potential, and promote improved aerobics courses' quality.

## 3. Methodology

### 3.1. Aerobics Posture Estimation Based on Inertial Sensor

The ZigBee wireless sensor network is responsible for collecting the data of the inertial sensors and transmitting it to the cloud platform via Ethernet. The cloud analyzes the data and inputs it to the BiLSTM network [24] for aerobics recognition. Because of different aerobics sports scenarios, a single estimation strategy cannot adapt to complex human movement patterns. Its diversified estimation strategies can fit the actual situation of human movement. The algorithm in this paper adopts dynamic strategies and steady-state strategies to correspond to different sports modes to increase the algorithm's efficiency, as shown in Figure 1.

Although Euler angles can more intuitively describe the posture of aerobics, there is a problem with gimbal locks. In addition, the quaternion method is more efficient to calculate, so this article uses rotating quaternion to describe any human body motion posture. Human pose estimation aims to find a rotating quaternion that can rotate any vector *x* in the limb coordinate system to the reference coordinate system. The following equation can express this rotation relationship:

(1) xR=qBR−1⊗Bx⊗qBR.

where ⊗ represents quaternion multiplication and (_*B*_^*R*^*q*)^−1^ is the inverse of the quaternion (_*B*_^*R*^*q*). In addition, in the field of attitude estimation, a typical somatosensory network needs to process data from multiple magnetic-inertial sensors at the same time.

The measurement signals of accelerometers and magnetometers can be divided into the following parts:

(2) $$\begin{array}{c} \left\{\begin{array}{c} S_{A}=g+b_{A}+n_{A},\\ S_{M}=m+b_{M}+n_{M}, \end{array}\right) \end{array}$$

where *g* is the gravitational acceleration, *m* is the strength of the Earth's magnetic field, *b*_*A*_ is the linear acceleration interference introduced due to human movement, *b*_*M*_ is the magnetic field interference generated by the ferromagnetic material in the environment, *n*_*A*_ and *n*_*M*_ are the sensors generated by the sensor measurement, respectively, noise can be simply assumed to be Gaussian white noise with zero mean.

The measurement equation of the gyroscope is as follows:

(3) $$\begin{array}{c} S_{G}=\omega +n_{G}, \end{array}$$

where *ω* is the angular velocity and *n*_*G*_ is the measured noise, which is considered to be Gaussian white noise with a mean value of zero.

### 3.2. Aerobics Action Recognition Based on BiLSTM

In this paper, a new neural network model [25–27] is constructed based on BiLSTM combined with adversarial training and attention mechanism. First, use BiLSTM to express contextual information more abundantly. Second, use the attention mechanism [28, 29] to calculate the importance of features, assign different weights to them, enhance the expression of features with the ability to distinguish categories, and weaken the influence of redundant features on the recognition of aerobics actions. Then, make a slight disturbance on the LSTM input layer through the loss function to verify the influence of the disturbance on the recognition of aerobics actions, and the model is shown in Figure 2.

Each sequence of BiLSTM has two LSTM layers: forward and backward, respectively, which makes up for the lack of contextual semantic information of LSTM. Each LSTM layer corresponds to an output layer. The bidirectional structure provides complete past and future context information at each moment in the input sequence of the output layer. The gate mechanism determines the transmission of information and can learn information that is important to current information. The forget gate determines which information is not important for classification. The input gate determines which information needs to be updated. The output gate determines which information to output; the state information of the hidden layer at a time *t* of the BiLSTM layer is updated as follows:

(4) $$\begin{array}{c} h^{t}=o_{t}e\;\tanh\left(C_{t}\right), \end{array}$$

where *h*^*t*^ is composed of forward *h*^*t*^ and backward *h*^*t*^ states and *W*_*f*_, *W*_*i*_, *W*_o_, and *W*_c_ are the forget gate, input gate, output gate, and updated weight, respectively.

The two functions of the attention mechanism are as follows: selecting the important information within the visual scope and reasonably arranging focusing visual resources to present the important information. Neural network attention mechanism can make the network model focus on the information input and then select the essential characteristics of the attention mechanism to accept any input. Regardless of its structure, under the condition of limited computing power, attention mechanism is the main method to solve information overload and a kind of effective resource allocation scheme; computing resources can be allocated to more important task information.

In the process of aerobics movement recognition, the traditional method directly sums up the updated output vector corresponding to each moment of the BiLSTM layer. It takes the average value so that it is assumed that each feature has the same contribution degree. However, feature vectors represent high-dimensional sparse features with a large number of noise and redundant features. Direct summing and averaging will easily lead to low classification accuracy. Therefore, we expect redundant or unimportant features to take a smaller proportion of weight. In comparison, features with a strong ability to distinguish categories will take a more significant proportion of weight.

In recent years, the attention mechanism has been applied to various recognition tasks [30, 31]. It is similar to the human brain's attention distribution mechanism. It quickly scans the scene in front of you through vision and focuses on the target scene that needs to be focused. Then, it takes a lot of this target scene time, and attention is used to obtain more detailed information related to the target scene, which in turn contradicts other useless information. The human attention mechanism dramatically improves the accuracy and efficiency of information processing in the visual range. In natural language processing text classification for reference, the attention mechanism is divided into different proportion weights for the areas with different contributions to the current task. The purpose is to filter out the more critical information for classification from a large amount of information, as shown in Figure 3. The attention mechanism coding model, the form of the attention mechanism distribution weight, is shown in the following equations:

(5) $$\begin{array}{c} u_{t}=\tanh\left(W_{w}h^{t}+b_{w}\right),\\ a^{t}=\frac{\exp\left(u_{t}^{T}u_{w}\right)}{\sum_{t}\exp\left(u_{t}^{T}u_{w}\right)}. \end{array}$$

Feed the two parts of the input layer to the model for training. After passing the BiLSTM layer and the attention mechanism layer, the cross-entropy loss function of the model is calculated through the softmax layer as shown in the following equations:

(6) $$\begin{array}{c} \text{loss}=\frac{1}{2}\left({\text{loss}}_{1}+{\text{loss}}_{a}\right),\\ {\text{loss}}_{1}=-\;\log\;p\left(y|x;\bar{\theta }\right),\\ {\text{loss}}_{a}=-\;\log\;p\left(y|x+r_{a};\bar{\theta }\right). \end{array}$$

## 4. Experiments and Results

### 4.1. Experimental Setup

This study selects 800 college students from a certain city as the research objects. According to their gender and aerobics level, they are divided into male, first-grade aerobics, male second-grade aerobics, male general, and female athletes. There was no statistical difference in basic information such as height, weight, and BMI for 10 people in each group, including the first-level female aerobics group, the second-level female aerobics group, and the female general student group.

The experimental environment configuration is Intel i5-3337U 1.8 GHz, 4G memory, Windows7 64-bit system. The experimental simulation uses a framework based on TensorFlow 1.9.0, and the programming language is implemented using Python 3.5 and MATLAB R2017b.

### 4.2. Experimental Result

Figures 4–7 show the recognition results of stepping, pony jumping, V-step, and walking in aerobics. The circle is the correct aerobics action category, and ^*∗*^ is the action category recognized by the model.

It can be seen from the above results that when performing action recognition on aerobics, recognition rates of 84.59%, 81.74%, 88.70%, and 85.22% were obtained, respectively, which proves the effectiveness of the model in this paper.

## 5. Conclusion

In this paper, a motion prediction model of aerobics athletes is built based on the wearable inertial sensor of the Internet of Things and the bidirectional long short term memory network. Firstly, a wireless sensor network based on ZigBee was designed and implemented to collect the posture data of aerobics athletes through inertial sensors. It transmits the data to the cloud platform through Ethernet. Then, the movement of aerobics athletes is recognized and predicted by the BiLSTM network. Based on the BISTM network and the attention mechanism, this paper proposes to solve the problem of low classification accuracy caused by the traditional method of directly summing and averaging the updated output vectors corresponding to each moment of the BiLSTM layer. The simulation experiment is also carried out in this paper. The experimental results show that the proposed model can recognize aerobics effectively. It enables students not only to learn the movement routines but also essential in learning the arrangement methods and leading exercises of high-quality courses. It constantly imitates and learns, finds the way and style suitable for their own, stimulates students' innovation ability, and promotes improved aerobics courses' quality.

## Figures and Tables

**Figure 1:** The block diagram of the approach based on IoT.

**Figure 2:** Aerobics recognition model.

**Figure 3:** Encoding model based on attention mechanism.

**Figure 4:** Recognition results of stepping.

**Figure 5:** Recognition results of pony jumping.

**Figure 6:** Recognition results of V-step.

**Figure 7:** Recognition results of walking.

## Data Availability

The data used to support the findings of this study are included within the article.
